# A Comprehensive Assessment of Cultivation Environment of Top Innovative High-Level Talents Based on Deep Learning Algorithm

**DOI:** 10.1155/2022/4846103

**Published:** 2022-09-19

**Authors:** Wei Zhu, Jin Qin

**Affiliations:** ^1^Office of Strategic Planning and Discipline Construction, Central South University, Changsha 410083, China; ^2^School of Resources and Safety Engineering, Central South University, Changsha 410083, China; ^3^School of Traffic and Transportation Engineering, Central South University, Changsha 410075, China

## Abstract

The quality of talent has increased across all fields due to the constant growth of different industries and the growing job saturation. Real-time job information on recruitment platforms can, therefore, accurately reflect the demand for talent from businesses, serving as a basis for the creation of training policies in schools. In international competition, the development of talents, especially top-level talents, will become more and more crucial. Growing in importance is China's economy and social development. The evaluation of higher vocational and technical talents, however, should also be assessed from a variety of angles, given the diversification of talent training objectives and teaching methods, as well as the expansion of teaching functions. An emerging machine learning technology called deep learning (DL) has been developed to bring machine learning closer to the goals of artificial intelligence. This essay offers a thorough evaluation of the depth of deep learning as it relates to the development of innovative talent in schools. The entire school must be strengthened. It is demonstrated that the average execution time is slashed by 0.0024 s, and the learning sample size error of the DL model is reduced by 0.05276 when compared to the Apriori method. As a result, implementing and researching the DL model can significantly improve both the overall teaching quality of schools and their capacity for innovation.

## 1. Introduction

Human resources with talents are those who possess specific professional knowledge or skills, engage in creative work, significantly improve society, and possess high ability and quality [1]. Cultivating new, high-quality manufacturing talent has become a crucial task to realize the construction of China's manufacturing power because new industries have brought about a new era of information technology, which has altered the demand for talents in this field [2]. Chinese schools now have a new mission to develop talents as a result of the advent of the “big data” era [3]. It is difficult for educators to adjust to the “big data” development trend and give students a better environment for learning and growth [4]. Schools are where the nation's future leaders will be trained, so society must plan for them in advance and understand what it needs based on the employment trends in each sector over the previous few years [5]. The development of the talent pool, especially the senior talent pool, will continue to gain importance in international competition and play a significant role in this process as one of the most significant influencing factors in the process of international production. Play a bigger and bigger role in the social and economic development of the country [6].

A dynamic system project called the Comprehensive Evaluation of the Quality of Advanced Personnel Training is based on the situations and tasks that talented individuals in higher education and scientific institutions perform in the real world. Utilizing cutting-edge technologies, extensive data collection, scientifically sound methods, evaluation of basic quality indicators, thorough ability and work performance of talents, inspection, evaluation, regulation, supervision, and implementation of education and scientific research, among other positions. The quality of Chinese higher education currently falls short of what is required for China's economic and social development, and the methods and indicators chosen to measure the effectiveness of talent development in schools have some flaws. It only serves as a static evaluation of particular assessment points and lacks any particular relevance. Despite being a sophisticated machine learning algorithm [7–9], DL has outperformed its forerunners in terms of speech and image recognition [10–12]. Therefore, meeting the demand for new, high-quality IT talent under the new social norm and promoting the close integration of educational “industry” and education are important tests for contemporary educators under the concept of “innovation-led.”

High-quality talents are the key resources for countries to take advantage of global competition, and the development of talents and human resources is more important than ever [13]. As a key institution for top-level talents education and training, schools should integrate resources, adjust the professional environment and structure according to the needs, and reform training programs as soon as possible according to the implementation of relevant national policies to meet the requirements [14]. In order to properly develop relevant and innovative specialties, pedagogy-related courses are integrated into training to achieve effective integration and coordination of science, engineering, and pedagogy to meet the needs of different aspects of society [15]. Pioneering innovation requires systematic analysis and study of talent training. Therefore, there is an urgent need to establish an effective quality evaluation system of talent training to guarantee the comprehensive reform of education.

The innovative points of this paper are as follows:

1. This thesis empirically analyzes the contribution of top-level talents supplemented by regional economic development laws to regional economic development and proposes countermeasures to cultivate top-level talents with certain realistic significance.
2. This study strengthens the management level of the top-level talents team in each school, enhances the core competitiveness of the school, guarantees the sustainable development of the school in the new era, and strengthens the field of higher education through this study.
3. This study has theoretical significance by investigating the current situation of advanced talents cultivation and exploring a unique cultivation mechanism that suits its own situation.

## 2. Related Work

### 2.1. Comprehensive Evaluation of Cultivation Quality of Top-Level Talents

As we enter the era of knowledge economy, the West has started to actively carry out research on talent and management. As a strategic project, China's future talent training operation should adhere to the policy of “service first, talent first, innovative mechanism, advanced leadership, and integrated development,” fully implement the strategy of strengthening the country with talents, and strengthen various functions. The formation of the modern development of the type of talent team, to accelerate the transformation of economic development, to achieve scientific progress to provide talent security.

Guo et al. investigated the employment matching degree of college students in the past 5 years through a multidimensional survey of the employment matching degree questionnaire of the majors studied and the initial employment [16]. Yang analyzed the problems of the top-level talents team and the defects of the talent incentive mechanism in the western region in order to improve and innovate the existing incentive mechanism and attract more foreign top to establish bases in the western region [17]. Wang concludes that there is a contradiction between school talents from a theoretical point of view, taking into account the real situation of the professional environment in 20 schools, the changes in local industrial restructuring, and job market demand in recent years. The training environment, the degree of matching with employment, and the working environment of schools are presented, recommended [18]. According to the characteristics of economic and social development, Fu et al. argued that “the top-level talents team of special industries is the key to promote the development of special economy and has an important demonstration and driving effect on the overall construction” [19]. Based on the proposed data mining and data analysis algorithms, Adribigbe's multidimensional career assessment model based on logistic regression and decision tree algorithms, an example of an assessment model that can be used to predict the quality of jobs to be fulfilled, is given. The use of the assessment model enables the prediction of occupational qualities that meet the common needs of vocational and personalized school graduates and helps to improve the quality of employment of graduates [20].

The government is currently in charge of evaluating the quality of talent cultivation in China, and it primarily gauges each school's educational standing by assessing the proficiency of its general school teachers. Due to the complexity and diversity of top-level talents, the comprehensive evaluation system of their cultivation quality typically contains a large number of unique indicators, making the process of comprehensive assessment's solution engineering challenging and complex.

### 2.2. Deep Learning Technology

The existing evaluation method is that experts give scores to each evaluation index, and then the final score of each talent is obtained by a simple weighted average, and the subjective factors of experts greatly affect the objective accuracy of the evaluation process and results. DL is a special kind of deep learning model. Many achievements have been made in search technology, data mining, machine learning, machine translation, natural language processing, multimedia learning, speech, recommendation and personalization technology, and other related fields.

After Zhang and Cao proposed the perceptron model, research on artificial neural networks began to increase, and there was a strong interest in this learning model of biological neural system models [21]. Terada and Watanobe trained deep neural network models with high-dimensional features after the introduction of deep neural networks with a complete representation of correlation information between features of sample data, combined with continuous feature information to form higher-order features and dimensional feature samples [22]. Doleck et al. proposed a novel feedforward network learning algorithm for solving large-scale linear equations based on the introduction of the conjugate gradient method [23]. The algorithm not only converges faster for optimal learning methods but also reduces the computational complexity of the method with better learning accuracy and better generalization prediction capability. Lin et al. later proposed a greedy algorithm for RBM, which trains layer by layer from the lower data input layer to the upper resultant output layer, treating the deep neural network as a combination of multiple layers before the conventional error backpropagation training. The difficulty of training deep neural networks was overcome by model pretraining [24]. Mara et al. proposed a matrix-based quadratic learning algorithm that can avoid the drawbacks of the standard algorithm, such as slow convergence and susceptibility to local minima, and overcome the disadvantages of computational complexity and large memory requirements [25].

Investing in human capital can bring greater returns than physical capital. The competition among world powers is no longer measured by the amount of raw material wealth but more by the competition for talent, especially top-level talents. Therefore, using deep models to learn features from large amounts of data can effectively engrave rich information into the data.

## 3. Comprehensive Evaluation of Training Quality of Top-Level Talents Based on DL Algorithm

### 3.1. Construction of Innovative Top-Level Talents Training Mode Based on DL

Top-level talents, who are responsible for the majority of the research on complex academic issues in educational institutions, see it as their duty to advance knowledge and innovate, and they place a premium on developing their own intellectual growth through academic research activities and honing their ability to reason logically [26]. High fault tolerance, self-learning capability, and parallel distributed processing [27] power are just a few of the characteristics of top-level talent cultivation models. Its distinctive knowledge representation and highly adaptive learning capacity have drawn significant interest from a range of subject areas. According to the own rules of talent growth and relevant influencing factors, and in accordance with the principles of scientific, operable, and comprehensive selection of evaluation indexes, the process of building a comprehensive evaluation index system for the cultivation of innovative talents in schools is depicted in Figure 1.

First of all, in the school innovative talent training system, the system operation must have the information goal, indicating the direction of the whole activity and the degree to be achieved, which is the training goal and training specification of the talent training system. The recruitment demand of enterprises is influenced by many factors and changes. In order to study the current situation of matching the demand for enterprise big data class jobs with the talent training of schools, we have to use python to obtain and preprocess the data of enterprise job demand and use the SARIMA-BP improvement model applicable to this scenario for modeling. It requires loading some binary code into each client and then converting the JDBC calls from the loaded client API to Oracle, Sybase, Informix, DB2, or other DBMS transfers. Thus given two point sets consisting of the following:

(1) $$\begin{array}{c} A=\left\{\left(A_{1},w\left(A_{1}\right),\left(A_{2},w\left(A_{2}\right)\right),\ldots ,\left(A_{m},w\left(A_{m}\right)\right)\right)\right\},\\ B=\left\{\left(B_{1},w\left(B_{1}\right),\left(B_{2},w\left(B_{2}\right)\right),\ldots ,\left(B_{m},w\left(B_{m}\right)\right)\right)\right\}, \end{array}$$

*w*(*A*_*i*_), *w*(*B*_*i*_), weight.

Students lack awareness at the level of consciousness of innovation education, are not clear about the meaning of innovation, and lack initiative and motivation for innovation education [28]. Therefore, school top-level talents should adhere to the independence of academic activities and should truly engage in research activities from the perspective of meeting the needs of society, rather than researching whatever is popular.

Secondly, according to cybernetics, the target information is not a signal and cannot act directly on the controlled object; it must go through the control mechanism and transform the training goals into executable information, which is the training program, including the curriculum and its structural form. As a result, the composition of the school's innovative talent training system is shown in Figure 2.

View autocorrelation and partial autocorrelation plots for model identification, and call the bic function to output BIC values to estimate model parameters to determine the model. The school innovation and entrepreneurship structure lack planned and systematic organization and management, setting up courses are superficial, and various events are neglected. The traditional approach is to use a measure of proximity, which in most cases is expressed as the sum of squared errors (SSE). The SSE is defined as follows:

(2) $$\begin{array}{c} \text{SSE}=\sum_{i=1}^{k}\sum_{\lambda \in c_{i}}\text{dis}\left(v_{i},x\right),\\ C_{i}=\frac{1}{m_{i}}\sum_{\lambda \in c_{i}}x, \end{array}$$

*m*_*i*_—the number of samples. *v*_*i*_—central point. *k*—cluster number. *x*—cluster sample. *c*_*i*_—class *i*.

The lack of benchmark student representatives in school innovation and entrepreneurship education has led to a serious lag in the overall educational mechanism and teaching effectiveness, and the effectiveness of education has been seriously affected [29]. If all layers of a deep network are trained simultaneously, the time complexity will be too high; if they are trained one layer at a time, the bias will be transmitted layer by layer. Neuronal models are commonly described by first-order differential equations, which can model the change of DL synaptic membrane potential with time:

(3) $$\begin{array}{c} \left\{\begin{array}{c} y_{i}\left(t\right)=f\left[u_{i}\left(t\right)\right],\\ \tau \frac{\text{d}u}{\text{d}t}=-u_{i}\left(t\right)+\sum w_{ij}x_{j}\left(t\right), \end{array}\right. \end{array}$$

*u*_*i*_—the internal state of neurons, *θ*—threshold value. *x*_*i*_—input signal.

At the same time, because deep networks have too many neurons and parameters, they face the opposite problem of supervised learning, where the data are severely underfitted. Thus, school top-level talents must insist on the purpose of research and the academic activity itself rather than just considering the effectiveness, and school top-level talents should see themselves as scholars first and teachers second, and only carry out independent research work and actively expand the boundaries of knowledge themselves to ensure the vitality of the school.

Finally, control signals must be transmitted along with the execution signal transmission to guarantee that the actuators and controlled objects overcome the impact of internal and external disturbances and can execute and receive execution signals in accordance with specific operation specifications. A set of rules and policies for managing teaching and education are the control signal in the talent training system. The SARIMA model's potential parameters can be predicted using the methods mentioned above, and the model can then be optimized using techniques like residual analysis and error evaluation, among others. The model needs to be adjusted and reestimated if the predicted value differs significantly from the actual value. If the difference is within an acceptable range, the prediction portion of the BP network can be used. The model will fit the survey data more accurately if the GFI and RMSEA values satisfy the model fitting requirements.

(4) $$\begin{array}{c} i_{t}=\sigma \left(W_{i}x_{t}+U_{i}h_{t}-1+V_{i}c_{t}-1+b_{i}\right), \end{array}$$

*i*_*t*_—input gate. *x*_*t*_—input data of the current time step (time t); *f*_*t*_—forgetting gate determines the retention degree of input data.

Top-level talents should adhere to both the scientific nature of research activities and the practical value of research in their research and academic activities. Top-level talents should ensure that their research activities can benefit society and consider the social impact caused by their research. The quality of innovative talent training involves a wide range of aspects and lacks a very scientific and objective assessment method. The operation of the talent cultivation model is a sustainable process, and the evaluation of milestones cannot reflect the real meaning of evaluation.

### 3.2. Establishment of Comprehensive Evaluation Index System for Talent Cultivation

Economic growth mainly relies on the investment of physical capital to achieve, but with the arrival of socialized mass production and knowledge-based economy, the investment of physical capital alone is far from satisfying the needs of social development [30]. The competition among world powers is no longer only measured by the amount of original material wealth but also by the competition of talents, especially the competition of top-level talents.

First and foremost, through management, we should establish an advanced education concept, make appropriate management policies that are conducive to mobilizing all parties, and establish a good campus atmosphere to create good environmental conditions for the cultivation of innovative talents. After clarifying the key components of the mechanism for cultivating top-level talents, we must be clear that the development of top-level talents is also influenced by a variety of factors. Personal factors primarily refer to an individual's efforts, psychological make-up, IQ, and other traits. The local perceptual area is used as the input to the lowest layer of the hierarchical structure in a convolutional neural network, and the information is transmitted to the various layers in turn, with each layer passing a digital filter to obtain the most important features of the observed data. The objective function can be chosen as follows when the Euclidean distance is used as the nonsimilarity index between the vectors in the group and the corresponding clustering centers:

(5) $$\begin{array}{c} J=\sum_{i=1}^{c}J_{i}=\sum_{i=1}^{c}\left({\sum_{k,x_{k}\in G_{i}}\left\|x_{k}-c_{i}\right\|}^{2}\right), \end{array}$$

*J*_*i*_—objective function.

This method is able to obtain salient features of the observed data that are invariant to translation, scaling, and rotation. The selection of variables is mainly based on the purpose of data mining. The variables that are closely related to the purpose of mining are selected, and it is required that the variables should not be highly correlated with each other. Otherwise, the mining effect will be affected.

Secondly, before data modeling, valid data needs to be prepared for modeling. Quality data is the basis for building a good model, and data preparation for modeling is done after the above data organization. Each time a sample R is randomly taken out from the training sample set, then the k nearest neighbor samples of R are found from the same kind of sample set as R, and then the weights of each feature are updated as the following equation:

(6) $$\begin{array}{c} W\left(A\right)=W\left(A\right)-\sum_{j=1}^{k}\text{diff}\left(A,R,H_{j}\right), \end{array}$$

diff(*A*, *R*, *H*_*j*_)—the difference between *R*_1_ and *R*_2_ in characteristic *A*;

Since the three-layer structure of the BP neural network can fit to approximate any desired nonlinear (or linear) continuous function with any desired accuracy, here, a three-layer BP neural network is used for quantitative analysis, and the three-layer BP neural network model is shown in Figure 3.

The development and formation of a top-level talent team can be assessed as follows: only the entire society exhibits respect for knowledge and talent, and societies and governments at all levels place a greater emphasis on education. The energy of the network decreases with increasing probability distribution concentration while increasing with decreasing probability distribution concentration. According to the philosophy of the multiple intelligence theory of human development, students' diversified intelligence should be fostered, and humanistic quality courses like those that develop students' communication and leadership skills and independent critical thinking skills should be incorporated into the curriculum system to form a curriculum system that fosters the objective of whole-person development. The following is assumed to be the reality of talent development in the school:

(7) $$\begin{array}{c} Ry=f\left(X_{1},X_{2},X_{3},X_{4}\right)\geq 0. \end{array}$$

The expected results are as follows:

(8) $$\begin{array}{c} Ey=f\left(\bar{X_{1}},\bar{X_{2}},\bar{X_{3}},\bar{X_{4}}\right)\geq 0. \end{array}$$

Then the difference between them is as follows:

(9) $$\begin{array}{c} D=\left\|Ey-Ry\right\|=\left\|f\left(\bar{X_{1}},\bar{X_{2}},\bar{X_{3}},\bar{X_{4}}\right)-f\left(X_{1},X_{2},X_{3},X_{4}\right)\right\|. \end{array}$$

In other words, the value of the energy function is lowest when the network is the most stable. By avoiding correlation and overlap between the original variables, the extracted few composite factors not only preserve the majority of the information from the original variables but also make them more representative and scientific. It is fair to say that factor analysis is a method for simplifying complex data because it can achieve the goal of “dimensionality reduction” by making the analysis problem less complex.

The time series model error is finally eliminated using BP neural network prediction, and the prediction data can be output to finish the combined model prediction when the error result is expected. It is critical to choose the initial weights and thresholds of the BP neural network in a sensible manner because they influence the network's convergence and make it simple to fall into a local optimum. In the BP neural network, the initial weights and thresholds play a crucial role. Thus, in accordance with the law of talent growth and associated influencing factors, we adhere to the principle of scientific, practicable, and comprehensive selection of evaluation indexes in order to fully reflect the current situation of top-level talents cultivation effect, fully exploit the human capital potential, further promote industrial upgrading, and achieve sustainable economic development.

## 4. Application and Analysis of DL Algorithm in Comprehensive Evaluation of Talent Training Quality

### 4.1. Initialization Analysis of DL

The initialization of the convolutional neural network is mainly to initialize the convolutional kernels and offsets of the convolutional and output layers and generally uses random initialization of the convolutional kernels (weighting), while the offsets are initialized with all zeros.

First, the residual in the convolutional neural network's output layer is calculated differently from its residual in the intermediate layer. The residual in the output layer is the difference between the output value and the class standard value, whereas the residual in the intermediate layer is obtained by weighted summing of the residuals in the following layer. Forward transmission involves transmitting the input signal from the hider to the output layer and producing the output signal there. It enters the error signal reverse transmission process if the output layer is unable to produce the expected output. The model takes user input and removes some scripting language in order to stop common script insertion behaviors that could impair the model's functionality and steal the user's data. This paper compares the DL-based and FNN-based approaches to verify the accuracy of the aforementioned two models. The results are shown in Figure 4.

The construction of special courses is an important part of the integrated curriculum construction of engineering education. According to its own characteristics and advantages, the school builds a number of disciplines that can play a leading and exemplary role in the curriculum system, teaching content, teachers' team, and teaching materials. With the construction of special courses to drive the development of other disciplines, the construction of special courses promotes the overall teaching quality of the school. Many factors such as network depth, convolutional kernel size, number of convolutional kernels, sample pool size, sample pool size, and location combine to affect the performance of the model. If a step is too far across, a large amount of curve information will be lost, resulting in partial linearization overload; it takes a longer time to get to the end of the curve because the span is too short. Therefore, it is important to consider the practical issues when choosing the learning speed. In the task creation based on the basic scheduling algorithm of Kubernetes, a set of test data that often occurs in the test was selected because of the great randomness of the task in selecting the target node, and the results are shown in Table 1.

Second, after the residuals are calculated for each level, the weights can be updated and adjusted, and the network performance is finally optimized after several training and adjustment sessions. Here, this parameter and bias cause the degree of nonlinearity of the Sigmoid function to change. If it has a low value, then it operates as a linear operation, and sampling is an example of patterning. If it has a large value, then the offset-based magnitude can be used as an “or” operation. Throughout the process, tests were performed in a fixed-point format, and the results were tallied and tested repeatedly in different data formats that were expressed in a narrower range and with less accuracy. The computational errors of the network in different numerical formats are shown in Figure 5.

However, the different statistical characteristics of the noise in the real environment lead to a significant impact of the edge distribution on the estimation of the original parameters, and also, the computational speed of the reduced noise autocoding algorithm is slower than other algorithms. In essence, it is a gradient-based fast decreasing method, which minimizes the final deviation by bootstrapping the first-order derivatives of the weights and explicating values.

The network weights are finally adjusted by error feedback when the error signal is transmitted backward from the output to the other layer, which improves system performance but at a relatively slow rate because the true output of the network is closer to the number of samples of the desired output. Smaller is not always better for a particular type of test target, and by testing two samples, we can find that the system performs better at 10∗10 and 15∗15. A scientific curriculum must be developed from the actual situation of schools and their training objectives because it is very challenging to make the fundamental quality of teachers and trainees in schools significantly improve in a short period of time. The sampling layer maps individual features onto a plane, whereas the convolution layer extracts local features. This technique can be used to determine the feature-to-feature location relationship with invariant displacement properties.

### 4.2. DL Training Process in Comprehensive Evaluation of Talent Training Quality

The DL algorithm is used to train the layered parameters in layers after achieving unsupervised training by using a bottom-up unsupervised learning approach or by building individual neurons layer by layer. The speed of training will significantly increase due to the network's rapid growth, and Figure 6 shows the iteration rate of model training before and after the Ceph distributed file system was optimized.

The talent cultivation input system, which is the precourse construction, is a thorough higher education talent cultivation resource. Its content includes the school's operating philosophy, financial investments, instruments and equipment, teaching materials, the team of teachers, the caliber of the students, professional structure, etc. It is a relatively stable factor that is directly related to the existing operational conditions of the school. The probability of discovery is slightly increased to increase the diversity of solutions, and it is slightly decreased during the final stage of the search to hasten the algorithm's convergence. Using 20 fuzzy criteria, the network's initial parameters were generated at random in [20, 50], and the identification Gabor function of DL was tested.

As can be seen from Table 2, with suitable initial fuzzy rules, the training sample error of DL is reduced by 0.05276, and the average running time is reduced by 0.0024 s compared with the Apriori algorithm, so DL has a good approximation effect.

Each layer in a convolutional neural network contains multiple neurons, and the neural units in the same feature graph share a single convolutional kernel or weighting. While convolutional kernels are a typical feature, if a convolutional kernel represents a curve, then the convolutional kernel will roll over the whole graph. The larger the amount of convolution, the more likely it is to be a curve.

Second, top-down supervised learning is used, i.e., a classifier is added to the topmost layer and the entire multilayer model is tuned using labeled data. Deep learning does not know the outside world, but it can view the tutor as an external knowledge expressed by feeding a set of output samples. We can also construct another kind of neural net (the structure here refers to the way neurons are connected to each other), i.e., a neural net containing many hidden layers. Maintaining the fortress also needs to be combined with network security measures such as network isolation and VPN to form a security audit space that is closed by the cloud security audit. The storage IO performance graphs before and after the virtualization build are shown in Figures 7 and 8.

The guidance signal or desired response shows the best results of deep learning. That is, it adjusts the network input so that the network output is close to the guidance signal or desired response. The type of deep learning algorithm depends on the variation of parameters, and each learning method has different advantages and adjusts the synaptic weights of neurons differently depending on the learning method. This refers to the various quality objectives set by the university according to its own management goals.

Finally, the number of neurons in the hidden layer is larger than the number of neurons in the input layer, and the self-writing method can be used to detect structural features. Usually, the convolutional and sampling layers are arranged alternately, in the order of convolutional, sampling, and convolutional layers. So the convolutional layers extract features from samples, then merge the samples to get more abstract features, and finally we get higher level image features. In this network structure, there are connections between neurons of the same level and restrictions between neurons, but it is still a feedforward network in terms of layer relationships.

## 5. Conclusions

The development of talents is a critical issue because they are necessary for the advancement of modern society. The initial emphasis on “elite education” has given way to a focus on “popularisation” in the higher education quality concept. A more recent issue is the demand for top-notch education for creative talent. The DL model is a network model with many hidden layers and a large number of data samples. The original data's information is directly input into the hidden layer, where the neuron nodes then automatically learn to enhance recognition performance. A sizable number of data samples and numerous hidden layers make up the network model. For the purpose of addressing the development requirements of China's high-level innovative nation, this paper proposes a thorough evaluation method based on the DL algorithm for the quality of top-level talent training in schools. Currently, the main problems with the comprehensive assessment system of top-level talent training quality in China are the current talent training system's shortcomings. The assessment and development of innovative talents in schools have been the subject of a fruitful discussion with the goal of promoting their growth and development. This is essential for developing the innovation system in Chinese schools.

## Figures and Tables

**Figure 1:** Build a comprehensive evaluation index system for innovative talents training in schools.

**Figure 2:** System diagram of innovative talents training.

**Figure 3:** Three-layer BP neural network model.

**Figure 4:** Comparison of fitting effects of two methods.

**Figure 5:** Network calculation errors in different numerical formats.

**Figure 6:** Comparison of the iterative speed of model training before and after optimization of Ceph distributed file system.

**Figure 7:** Storage IO performance chart before school virtualization construction.

**Figure 8:** Storage IO performance diagram after school virtualization construction.

**Table 1:** Comprehensive evaluation of task operation.

Task name	Running time		
	Model training (h)	Data processing (h)	Data annotation (h)
The AI basic scheduling algorithm is not used	6.54	1.34	7.32
Use AI basic scheduling method	2.51	3.23	4.64

**Table 2:** Experimental results of identifying Gabor function.

Algorithm	DL	Apriori
Training steps	14000	13000
Training sample error	0.00171	0.05447
Average running time per step (s)	0.0054	0.0078

## Data Availability

The data used to support the findings of this study are available from the corresponding author upon request.
